The article "On the Problems and Countermeasures of College Students' Mental Health and Safe Work under Network Environment" was retracted in 2023. Reasons: signs of a paper mill; suspected computer-generated content; unreliable results or conclusions; concerns about the data.

# On the Problems and Countermeasures of College Students' Mental Health and Safe Work under Network Environment

**DOI:** 10.1155/2022/2993982

**Published:** 2022-08-05

**Authors:** Yuanyuan Xu, Shuchao Liu, Yongdong Chen

**Affiliations:** ^1^School of Marxism, Chongqing Jiaotong University, Chongqing 400074, China; ^2^Office of Science and Technology, Chongqing Jiaotong University, Chongqing 400074, China; ^3^College of Electrical Engineering, Sichuan University, Chengdu 610044, China

## Abstract

Under the network environment, mental health and safety work on college is related to national security and campus security. Moreover, it affects the healthy development of college students. In the era of ever-changing mobile Internet, colleges and universities must take practical countermeasures against the problems in mental health and safety education on college and improve the relevance and effectiveness of college students' network safety education. This paper first finds the problems of college students' mental health and safety through questionnaire survey and analyzes the current situation of college students' mental health and safety under the current networked environment. In response to the problems found, we propose complete and systematic educational countermeasures. At the same time, we need to firmly establish the strategic awareness of network security education and strengthen the construction of network security education in colleges and universities. We should strengthen the construction of network security education in colleges and universities, form a joint effort of schools, families, government, and society, and improve the quality and effectiveness of network security education.

## 1. Introduction

Mental health is the foundation of talent quality, and only with a healthy psychology can the moral, intellectual, physical, and aesthetic development of college students be comprehensive [1]. Only with a healthy psychology can we cultivate the practical ability and innovative spirit of college students. As a special group, college students are in the process of maturity in psychological and physical aspects. During this period, they are more likely to have a series of physiological and psychological problems. If college students cannot adapt to the changes in study, life, and employment at this stage, they are more likely to have adverse effects on the psychological level [2]. If the adverse psychological effects are not taken seriously and solved in time, this will affect their study and life in college and even their work and life in the future. At the same time, due to the continuous development of higher education in China and the expansion of enrollment scale, the education management task of college students is getting more and heavier. Then, how to effectively conduct comprehensive and objective statistics on the mental health condition of college students so as to promote better mental health education of college students is urgent [3].

The article "On the Problems and Countermeasures of College Students' Mental Health and Safe Work under Network Environment" was retracted in 2023. Reasons: signs of a paper mill; suspected computer-generated content; unreliable results or conclusions; concerns about the data.

Network is a double-edged sword; with the development of mobile network information more and more rapidly, network security ferments rapidly. In recent years, network security incidents have often occurred in colleges and universities, which not only seriously affect students' daily life and psychological health but also threaten students' life and property safety [4]. At the present stage, many college students' network security awareness is relatively weak, their ability to deal with network emergencies is not strong, and they are easily influenced by the network environment [5]. Therefore, it is necessary to build students' awareness of network security in order to ensure the safety of college campus. At the present stage, college campuses are mainly for the “00” postgraduates who have just come of age, and their ability to judge and discern many things still needs to be improved. Cyberspace has the characteristics of interactivity and virtuality. At the same time, it is also a hotbed for many unscrupulous elements to work around and publish all kinds of bad information. As some college students have not received systematic and comprehensive education, they are easily deceived, which is not conducive to the healthy growth of college students [6].

With the increasing informatization of the society, the daily life of college students has been closely connected with the Internet and cannot be separated from it [7]. This group gradually occupies the network space and becomes the most active part, and they show their own behavioral characteristics when using the network. Throughout the group of college students, most of them have safe, positive, and healthy behaviors on the Internet. However, there is a small group of people whose online behavior violates the social norms of behavior, which has a negative impact and even hinders the way of college students' growth and adulthood [8]. In such a background where the Internet is becoming more and more closely related to reality, if such bad Internet behavior cannot be effectively stopped and solved, it will definitely cause great harm to the college students, the school, and even the national society. While the Internet brings endless convenience to college students, it is also a risky vortex for college students to be involved in Internet fraud, Internet addiction, Internet violence, and Internet infiltration. In order to reduce the harm brought to college students by network problems, network safety education must be on the agenda [9].

The article "On the Problems and Countermeasures of College Students' Mental Health and Safe Work under Network Environment" was retracted in 2023. Reasons: signs of a paper mill; suspected computer-generated content; unreliable results or conclusions; concerns about the data.

This paper takes the network environment as the research background and focuses on the problems and countermeasures of college students' mental health and safety work. Through the analysis of the current situation of college students' mental health in the network environment, the key problems of mental health and safety work are identified, which makes the mental health and safety education work more targeted and effective. Through the questionnaire survey, combined with theoretical research, the specific problems of college students' safety in the network environment are explored. The reasons affecting the effectiveness of safety education for college students are analyzed, and the focus is on exploring the path of improving network safety education. It also proposes educational countermeasures for mental health and safety issues on college in the network environment. This motivates college administrators, mental health teachers, and educators to pay more attention to creating a good network environment. It also suggests effective ways to strengthen values learning, will cultivation, and good moral behavior to college students from the side, so as to reduce the harm caused by the network environment to college students' mental health.

This paper consists of five main parts: the first part is the introduction, the second part is the state of the art, the third part is methodology, the fourth part is result analysis and discussion, and the fifth part is the conclusion.

## 2. State of the Art

### 2.1. Concept and Characteristics of the Network Environment

#### 2.1.1. The Concept of Network Environment

In a narrow sense, the network environment refers to a broadband, high-speed, integrated, wide-area digital telecommunication network built on the basis of the combination of electronic computers and modern communication technology [10]. This kind of network can cover one country, several countries, and even the whole world by setting up a network within a network and international interconnection. In a broader sense, the network environment also includes changes in national information policy, information management system, information system organization, user behavior, and social culture caused by network penetration and expansion. The former refers to the material entity of the network, which we may call the hardware of the network. The latter refers to the mental body (or abstract body) of the network, and we may call it the software of the network. The network environment of the information society should be a whole that contains both hardware and software. It includes not only network resources and network tools but also nonphysical forms such as learning atmosphere, learners' motivation, interpersonal relationships, and teaching strategies.

The article "On the Problems and Countermeasures of College Students' Mental Health and Safe Work under Network Environment" was retracted in 2023. Reasons: signs of a paper mill; suspected computer-generated content; unreliable results or conclusions; concerns about the data.

#### 2.1.2. Characteristics of the Network Environment

*(1) Resourcefulness and Share Ability*. The network connects information owners around the world through certain technologies and communication rules [11]. It achieves the maximization of network resources. The Internet has become the world's richest “library” of information by connecting various computer terminals. Anyone can get all kinds of information about human current affairs, news, culture, education, life, and so forth with a click of a mouse and truly “know everything without going home.” Most of the information on the Internet is free, and some of it is paid. But, no matter what way, the richness and sharing of network resources are attracting more and more people to use the network. As long as there is a network, people can upload all kinds of information to various platforms, and different people can download any resource through the network and publish it in their circle of friends. The information is circulated among different people to achieve resource sharing and improve the utilization rate of resources. It also demonstrates the richness and share ability of network resources.

*(2) Openness and Globalization*. As an information space, the network is composed of network hardware and network software. It does not belong to any one country, any one organization, any one nation, or even any one person. It is an open global system. Anyone can access any website around the world, browse information, exchange ideas, and so forth freely across time, space, race, gender, status, and age. Although different countries have their own cultural backgrounds, the spread of new things fully reflects the openness and global nature of the network.

*(3) Timeliness and Serviceability*. Nowadays, with the common use of smart phones, people are used to getting resources from the Internet. This requires that the delivery of information must be timely. Newspapers, TV, and other traditional media retain traditional communication methods and have opened synchronous electronic news on the Internet. Many major events are uploaded to the Internet by witnesses through cell phones and computers as soon as they happen. The audience can get the information and express their opinions at the same time. Through the Internet, people can interact with each other anytime and anywhere to speed up the spread of information. In the virtual society, people can chat, play games, entertain themselves, or shop, all of which are to meet the most basic needs of human beings. Fundamentally, the Internet has a social function of service, a way of service. The Internet connects more people and groups, providing them with various needs and satisfying their service requirements in various aspects.

The article "On the Problems and Countermeasures of College Students' Mental Health and Safe Work under Network Environment" was retracted in 2023. Reasons: signs of a paper mill; suspected computer-generated content; unreliable results or conclusions; concerns about the data.

### 2.2. Domestic and Foreign Research on Network Security

#### 2.2.1. Status of Domestic Research

Domestic research on personal factors of college students can be broadly divided into two aspects: personal basic conditions and psychological factors. Most of the studies on personal conditions are qualitative studies on the differences of college students' network safety perceptions in terms of gender, education, and major by using questionnaire surveys. According to the analysis results of the questionnaire survey conducted by literature [12] on college students, according to different sample types, male students, public security students, and engineering students would choose safer ways to pay and receive emails online. In the survey of Wuhan colleges and universities, it was found that the cognition of online security was more influenced by gender, education, and professional nature, and male students were stronger than female students, undergraduate students were stronger than graduate students, and academic students were stronger than technical students [13]. In terms of the difference in the cognitive ability of Internet fraud, the literature [14] found that the proportion of female college students being cheated was significantly higher than that of male college students when comparing college students of different genders encountering Internet fraud. The fact that female students are more likely to be cheated than male students indicates that female students are less able to recognize online frauds.

Relatively little research has been conducted on the psychological aspects of individuals, which are generally mentioned in studies of Internet addiction. The literature [15] suggests that Internet addictive behaviors are related to individual psychological characteristics, such as social fear, lack of self-confidence, depression, anxiety, and loneliness. The literature [16] found that the real-life loneliness of college students was predictive of the tendency to Internet addiction by studying the loneliness of college students and Internet addiction.

#### 2.2.2. Current Status of Foreign Research

From the research accounts of foreign scholars, it is generally believed that, based on the current development perspective of globalization and internationalization, it is still impossible for any country or region to control the network development trend. The literature [17] argues that the key factor in preventing network security risks is user behavior rather than technology. The literature [18] mentions that some countries in the EU integrate the content of cybersecurity education courses with psychology courses and social practice courses to make the content of cybersecurity education courses richer and more vivid. The literature [19] suggests that cybersecurity education courses should be incorporated into the existing curriculum system of universities to make cybersecurity education courses more formalized and standardized. Literature [20] mentions that the content of network safety education in American universities includes teaching students how to surf the Internet safely and how to protect their privacy. From the existing studies, it can be seen that the curriculum of network safety education in western countries has become a relatively complete system.

The article "On the Problems and Countermeasures of College Students' Mental Health and Safe Work under Network Environment" was retracted in 2023. Reasons: signs of a paper mill; suspected computer-generated content; unreliable results or conclusions; concerns about the data.

Many countermeasures have been proposed in foreign studies to educate college students about cybersecurity awareness. The literature [21] found that foreign college students face the risk of identity theft through fraudulent emails, stolen passwords, and unsafe online practices. Literature [9] suggests that female college students have become vulnerable to cybersecurity problems due to their physical and psychological characteristics, and more attention needs to be paid to their cybersecurity education.

## 3. Methodology

### 3.1. Problems and Causes of College Students' Mental Health

#### 3.1.1. Problems of College Students' Mental Health in the Network Environment

*(1) Blindness in Self-Perception and Evaluation*. The awareness of college students about the Internet is mainly at the level of use. They know very little about the mechanism of information dissemination and the social role of the Internet. Students are usually blind and vague about the multiple influences of the Internet and their purposes of accessing the Internet. Their Internet use behavior is basically spontaneous, and the supervision of school, family, and society is in a relative vacuum. In the traditional social environment, people's behaviors are often conscious, purposeful, controllable, and measurable. In contrast, college students appear to be blind in self-awareness evaluation in the network psychology, and they usually lack clear cognition about their social role positioning.

*(2) Utilitarianism of Value Orientation*. In the network environment, everything seems relatively virtual. Because of this, college students who use the Internet are satisfied with the virtual sense and the sensory enjoyment and life value affirmation obtained from the network environment. At the same time, a series of value drifting problems have emerged in this era, such as money worship, individualism, and anarchism which are very prominent. This makes college students have serious deviation in life values. They choose blindly in their beliefs, are at a loss in their life planning, and become more secularized and utilitarian in their lifestyles.

*(3) Vulgarization of Moral Outlook*. In the network environment, the space is virtual, the identity is hidden, and the restraint is weak. This makes college students reduce their control over their sense of responsibility. In the network environment, some college students show the dark side of human nature, moral indifference, and deviation from moral behavior, as well as reduced sense of moral responsibility. In other words, the Internet has encouraged their rebellious side. This directly leads some college students to form vulgar moral views and their human ecology begins to become somewhat “game state.” Their concern and sense of responsibility for their studies, future, and society are far from enough.

The article "On the Problems and Countermeasures of College Students' Mental Health and Safe Work under Network Environment" was retracted in 2023. Reasons: signs of a paper mill; suspected computer-generated content; unreliable results or conclusions; concerns about the data.

#### 3.1.2. Causes of Mental Health Problems among College Students

*(1) The Conflict between the Reality and the Virtual Nature of the Internet*. The Internet is a mapping of reality, but it cannot replace reality. Some college students with unhealthy psychological tendency cannot distinguish the difference between the network world and the real world. In their opinion, the network is life. Due to their upbringing, personality, and interests, they are reluctant to communicate with their classmates and teachers in face-to-face verbal communication. They tend to accumulate such negative emotions and energy in their subconscious, thus creating various psychological disorders or unhealthy psychological tendencies. The Internet, however, opens a virtual door for them and provides them with a mental haven. In their view, boredom, pain, anxiety, and other emotions can be released through cyberspace in the online environment. However, no matter what kind of pleasure they get in the online environment, the problems that exist in reality cannot be solved accordingly. After going offline, they still have to face these real psychological problems, and the sense of loss and alienation will become stronger and stronger. Out of avoidance, they will come into cyberspace again to seek solutions. Once this vicious circle accumulates to a certain extent, it will lead to serious psychological disorders.

*(2) The Conflict between Emotional Catharsis and Self-Control Out of Control*. According to the research findings, even those college students with excellent grades, outstanding appearance, and superior economic conditions would like to go to the cyberspace to find a larger range of recognition, respect, and spiritual support. In the online environment, people from different countries, races, and ways of thinking come together to create a broad stage for performance. In the cyberspace, college students can temporarily forget about their social roles, social influences, and face problems and express themselves as they like. What is more, some college students use network control to express their existence and value. Some college students who are proficient in network attack techniques often lose self-control in the process of emotional catharsis, causing serious infringement on the interests of others and society and moreover posing an objective threat to the network world.

*(3) The Conflict between Personality Factors and Internet Addiction*. College students with poor self-restraint ability are easily affected by the negative influence of the Internet. Those college students who pay attention to the present enjoyment are prone to the symptoms of Internet addiction. Those college students who care more about whether they accomplish their set goals can generally show stronger self-control in front of the Internet. Those who are frustrated, such as losing at work, social fears, or losing love, indulge in the Internet in order to seek relief and can rely on online stimulation to make up for the unsatisfied trauma of the oral period. The Internet becomes a mental agitator, a facilitator of secondary benefits, and a place for the realization of the spirit of entertainment supremacy.

The article "On the Problems and Countermeasures of College Students' Mental Health and Safe Work under Network Environment" was retracted in 2023. Reasons: signs of a paper mill; suspected computer-generated content; unreliable results or conclusions; concerns about the data.

### 3.2. Problems of College Students' Network Security Education

#### 3.2.1. Weak Awareness of Network Security

*(1) Weak Awareness of Privacy Protection*. The subject of privacy is a natural person, and the content of privacy refers to the fact or behavior that a specific person keeps secret about his affairs, information, or fields and does not want others to know or interfere in. According to the survey results, most college students are not aware of the protection of privacy contents such as name, ID number, and cell phone number. When asked “when you register a new account, which of the following information will you disclose or fill in?,” 26.79% of college students chose to fill in their name and year of birth. 45.01% of college students think they can disclose QQ, WeChat, and cell phone number. 14.43% of college students choose to fill in gender, ethnicity, and home address. 8.46% choose to fill in student ID, ID card, and graduation number. 5.31% choose to upload photos. Due to the technical loopholes of APP, students should fill in personal information selectively when seeking services through APP, such as cell phone number, home address, ID card number, student ID card, and graduation number, and photos should be added carefully. The specific situation is shown in Figure 1.

The article "On the Problems and Countermeasures of College Students' Mental Health and Safe Work under Network Environment" was retracted in 2023. Reasons: signs of a paper mill; suspected computer-generated content; unreliable results or conclusions; concerns about the data.

In response to the question “do you read the privacy policy when you register as a new user?,” 32.13% of college students chose “I don't read it carefully and I do n't think it's necessary.” 59.56% of the students said “I don't read it carefully, and I just read it in general.” 8.31% of the students chose “I will read it carefully.” According to the questionnaire data, students who “just read it” did not see any substantive content of the privacy policy but just skimmed a few times. The privacy policy is an electronic contract of use, which specifies your rights and obligations. However, the majority of college students does not see or even read the privacy policy, and their awareness of privacy protection is weak, which makes education about Internet security more difficult. The specific findings are shown in Figure 2.

*(2) Low Legal Consciousness*. According to the survey results, most college students have low legal literacy and weak legal awareness. When asked “which of the following incidents have you done?,” 7.71% of college students have used other people's articles and viewed other people's privacy without their consent. 51.26% of college students have used software to crack other people's WiFi password. 4.94% of college students have uploaded other people's photos or images privately. 2.43% of college students have used other people's names to do something against morality or even law. 6.47% of college students have viewed other people's cell phones, tablets, and computers without their consent. From the legal point of view, breaking others' WiFi passwords is suspected of violating others' personal property. The specific survey results are shown in Figure 3.

When asked “when you or your classmates encounter online fraud, how would you handle it?,” 27.82% of the students chose to report to the public security authorities to protect their own rights and interests by applying the relevant laws. 14.06% of the students would report to their class cadres and counselors in time. Meanwhile 28.63% of the students thought that if the amount was not large, they would admit their own bad luck and would not bother to deal with it. 6.81% of the students chose other ways to deal with it, while 22.68% had not encountered online fraud. The specific survey results are shown in Figure 4.

*(3) Weak Awareness of Protection*. With the advent of the Internet era, our living space has been greatly expanded. The “Internet+” has given birth to a new development model. The Internet is a “double-edged sword”; the popularity of the Internet not only brings convenience to the public at the same time but also gives rise to a series of security issues. They include system paralysis, hacker attacks, business leaks, network fraud, and privacy leaks.

The article "On the Problems and Countermeasures of College Students' Mental Health and Safe Work under Network Environment" was retracted in 2023. Reasons: signs of a paper mill; suspected computer-generated content; unreliable results or conclusions; concerns about the data.

In response to the question “what are the main software you use now for network security?,” 83.32% of college students chose “antivirus software.” 56.65% of college students chose “firewall.” 28.22% of the students chose “information content filtering,” and 26.04% chose “intrusion vulnerability checking.” 9.25% of the students chose “other.” When asked “do you know how to use firewall and antivirus software?” 16.92% of college students chose “yes and can operate it skillfully.” 65.65% of college students chose “half know” and 17.43% chose “no know.” The specific survey results are shown in Figures 5 and 6.

*(4) Low Discriminatory Ability of Network Information*. With the advent of the era of big data, the trend of explosive growth of Internet information has emerged. How to absorb the nutrients in the infinite network information and become a more qualified successor requires the contemporary college students to have a strong ability to distinguish the network information.

When asked “what would you do if you are asked to scan the QR code when you encounter a discount event?,” 9.57% of the college students often scan the QR code and think the security problem is not big. 62.39% of the college students choose to do it occasionally and are a bit worried about the security problem. 28.04% of the college students are very cautious and never scan it. The survey results show that most college students have the awareness of distinguishing online information, and only a few of them choose profit and give up online security when they are tempted by profit. However, only a few of them have the ability to distinguish online information among the majority of college students who have the awareness of distinguishing online information. The specific survey results are shown in Figure 7.

In response to the question “how would you choose to log in to the website provided by the recipient for the normal use of your bank card when you receive a text message?,” 28.64% of college students would check carefully before deciding whether to log in. 33.53% of the students thought it might be a phishing website and were vigilant about it. 4.81% of the students chose to wait and see if they would call the police. 33.02% of the students did not pay attention to it. The survey results show that two-thirds of college students have the awareness of discriminating online information when it is related to their own property security. Since college students come from different social environments before receiving higher education, they make choices with relative discernment under the guidance of discernment awareness. However, the remaining one-third of college students choose to ignore it and put their own property security in the online world indifferently, laying a hidden danger for the future network security problems. The specific survey results are shown in Figure 8.

*(5) Weak Self-Control Ability on the Internet*. With the further development of the information age, the Internet has become an indispensable means and carrier for college students' daily life, study, and communication with its rich content, fast transmission speed, and strong penetration. When asked “have you ever browsed unhealthy websites of pornography, gambling and drugs?,” it was found that 5.62% of college students often browse “pornographic, gambling and drug” websites. 36.54% of college students occasionally browse “pornographic, gambling and drug” websites. 57.84% of college students never browse “pornographic, gambling and drug” websites. The Internet economy is also known as the eyeball economy, and pornography, gambling, and drugs are wearing a bright veneer, occupying the sight of college students and eating up the world of college students. The specific survey results are shown in Figure 9.

The article "On the Problems and Countermeasures of College Students' Mental Health and Safe Work under Network Environment" was retracted in 2023. Reasons: signs of a paper mill; suspected computer-generated content; unreliable results or conclusions; concerns about the data.

#### 3.2.2. Inadequate Content of Network Security Education

Educational content refers to the overall culture of knowledge, skills, behavioral norms, values, and worldviews that are selected and incorporated into the process of educational activities in order to achieve educational goals. Network safety education is an educational activity to improve the comprehensive quality of college students to cope with the network society. The goal is to promote the all-round development of college students in both spaces. In order to achieve the goal of network safety education, scientific and reasonable lesson contents need to be selected.

*(1) Lack of Systematization of Education Content*. At present, the network security education in China's colleges and universities mainly relies on ideological and political education theory courses and public courses of college students' computer for realization. According to the attributes of disciplines, each discipline has its own educational goal, and the main purpose of college students' safety education is to improve college students' ability to cope with real-world safety. However, the content of network security education set by universities to achieve the educational objectives is mostly a simple superposition of the educational content of Civics and Political Science class, computer education content, and security education content. This leads to incomplete coverage of cybersecurity education content, lack of logic between education content and unsystematic structure of education content, and difficulty in achieving the optimal trend of education results.

*(2) Lack of Empathy in Education Content*. Education is a practical activity that affects students, and it is an art that touches students' emotions. In order to achieve a deep-rooted educational effect, it is necessary to build a sympathetic content system according to the needs of students. When asked “what aspects of network security education do you want to carry out?,” 62.39% of college students chose “basic computer knowledge.” 71.74% of college students chose “education on network security ethics and laws.” 58.61% of college students chose “education on network psychological health.” 36.76% of college students chose “education on mainstream ideology.” 3.18% of the students chose “other.” Among the other options, the participating college students also mentioned “education on online payment” and “prevention of online fraud.” The specific survey results are shown in Figure 10.

The article "On the Problems and Countermeasures of College Students' Mental Health and Safe Work under Network Environment" was retracted in 2023. Reasons: signs of a paper mill; suspected computer-generated content; unreliable results or conclusions; concerns about the data.

#### 3.2.3. School Teachers Do Not Pay Attention to Network Security Education

Colleges and universities are the main position of ideological and political education in China. Therefore, ideological and political educators play an irreplaceable role in the process of educating people. With the expansion of the virtual world, network safety education has become an important part of ideological and political education. Most of the network safety education activities in colleges and universities are organized by ideological and political educators, and the traditional safety education methods are mostly used in network safety education. These include classroom learning, expert lectures, window banners, club activities, and other methods. Under the guidance of traditional education methods, the survey results show that 13.86% of college students choose “great.” 61.42% of college students choose “average.” 18.47% of college students think it has little impact. 6.25% of college students choose “no impact.” At the same time, the survey results show that the impact of network security education in colleges and universities does not call for optimism. Although most colleges and universities carry out network security education, and the depth and breadth of the impact of network security education are worth our reflection. The specific survey results are shown in Figure 11.

## 4. Result Analysis and Discussion

### 4.1. Methods of Implementing Mental Health Education

The path of psychological education for college students in the network environment mainly revolves around the network, and the methods of mental health education for college students are innovated through the network. There are many forms of online psychological education activities, such as online psychological classroom, mental health public platform, class blog, mental health QQ group, and mental health education software. These activities are carried out by making full use of the Internet, which is a convenient and familiar way for college students to transmit mental health knowledge, contents, methods, and ideas. Through the development of various network psychological education activities, not only can college students fully experience the convenience brought by the progress of network technology, but also they establish the correct concept of mental health and guide their healthy psychological development through the development of activities. For example, online psychological classes can allow college students to communicate with specified experts and scholars thousands of miles away to solve their psychological confusion.

The article "On the Problems and Countermeasures of College Students' Mental Health and Safe Work under Network Environment" was retracted in 2023. Reasons: signs of a paper mill; suspected computer-generated content; unreliable results or conclusions; concerns about the data.

#### 4.1.1. Email

Colleges and universities can disclose the emails of psychological education and counseling workers to college students and inform them that they can contact them by e-mail to seek solutions to their psychological problems and confusions. The psychological educators who receive the emails should answer the students' questions in a timely manner to help them form a sound psychological concept of themselves and their ability to adapt to the outside world. At the same time, it should be noted that the student's identity and personal information should not be revealed. E-mail counseling is the best way to address sensitive issues such as sexual orientation, love, and psychological crime.

#### 4.1.2. Message Board

Leaving a message on the message board of psychological education forum is also a way to solve the psychological problems and confusion of college students. At present, BBS and public platform have become the network space that college students pay attention to, which makes it an important platform for psychological health education in colleges and universities. On this platform, colleges and universities can ask famous psychologists to solve college students' psychological problems.

#### 4.1.3. Internet Chatting Consultation

This is a kind of instant information exchange method, which is obviously different from the first two types of methods, and it requires experts or psychological educators to be on duty at a fixed period of time. Chatting can be done through QQ, WeChat, and MSN or in a special chat room, and the chat can be divided into text chat and voice chat. Due to the immediacy of information transmission, the effect of text chat is much stronger than traditional letter counseling, while voice counseling has a The part “Fourth, network conference counseling” is grammatically unclear. Please rephrase this part for clarity.better intervention effect on certain college students' psychological crisis.

The article "On the Problems and Countermeasures of College Students' Mental Health and Safe Work under Network Environment" was retracted in 2023. Reasons: signs of a paper mill; suspected computer-generated content; unreliable results or conclusions; concerns about the data.

#### 4.1.4. Web Conference Consultation

The most important feature of network conference is that it can use camera technology to allow experts and workers to talk with college students face to face. It is possible to judge the mental health condition of college students from their most intuitive visual perceptions such as voice, intonation, facial expressions, and body movements through the network technology. At the same time, the network meeting also breaks the limitation of time and geography, which makes the exchange and interaction of information possible. Although this is a relatively expensive way now, it will benefit many college students' mental health education as technology advances.

### 4.2. Strengthen the Governance of Cyberspace and Network Content Construction

First, the governance of cyberspace is strengthened to create a good network environment. The governance of cyberspace fundamentally lies in the strengthening of network legislation. At present, China's network legislation obviously lags behind the development speed of Internet technology, and the laws and regulations governing the network environment need to be improved. On the one hand, the network legislation is strengthened, and the principle of network access is regulated. For the practice of spreading network rumors, speculation, smearing historical figures, and spreading reactionary speech, we should increase the crackdown and punishment and severely pursue their legal responsibility. On the other hand, the control of network information is strengthened, and a clear mechanism of network supervision is established. The online behavior of online social platforms, online forums, and large websites is regulated.

Second, the construction of network content is strengthened, and the quality of network communication is improved. On the one hand, the top-level design is strengthened, and the network content is optimized. On the other hand, in the way of network content dissemination, the construction of network discourse system is strengthened, and the high ground of network propaganda is seized. Online ideological propaganda work to pay attention to the scientific and accurate network language. In addition, because ideological propaganda work is highly theoretical and is not easy to be understood and accepted by ordinary Internet users, we should use the Internet users to enjoy the dissemination, as well as innovative means of communication and popular language for explanation.

The article "On the Problems and Countermeasures of College Students' Mental Health and Safe Work under Network Environment" was retracted in 2023. Reasons: signs of a paper mill; suspected computer-generated content; unreliable results or conclusions; concerns about the data.

### 4.3. Strengthen the Construction of Campus Activities and Campus Culture

The good or bad campus environment is directly related to the effect of ideological safety education of college students. Campus culture is a microcosm of social life and campus life, and colleges and universities make use of the subtle inculcation and infection effect of culture on people. By improving campus cultural facilities, using campus media, and creating campus cultural activities, we can transmit the mainstream social values and ideology to students, so that their daily behavioral practices can truly conform to social standards and moral codes.

First of all, the construction of campus cultural facilities is strengthened and a good physical culture environment is built. Campus cultural facilities are the external expression of campus culture and the material carrier of campus culture construction. Universities should increase the investment in the construction of cultural facilities and make full use of campus radio stations, electronic displays, official websites, physical landscapes, and propaganda slogans to promote mainstream culture and mainstream ideology. We should make full use of the cultural facilities and educational functions of the campus, so that students can be influenced by the campus culture.

Second, the guidance function of campus media is strengthened. Campus media is an important position of school ideology and propaganda work and is an important channel for information transmission and ideological leadership. Campus media mainly includes campus radio stations, campus forums, school magazines and newspapers, official microblogs, and Weibo. Campus media propaganda work adheres to the correct value orientation and directional principles and strictly filters junk information and reactionary speech. Sensitive issues should be treated seriously and handled seriously to strengthen the dissemination of mainstream ideology among the student body.

### 4.4. Carry Out Legal Education and Raise Awareness of the Rule of Law

First, the education of legal knowledge of network security is strengthened, so that college students know the law and understand the law. Strengthening the network legal education of college students is an important link in the process of promoting the comprehensive rule of law. To strengthen the network legal education of college students, the first thing is to clarify the main content of network legal education. On the basis of clear education content, colleges and universities should offer the legal knowledge course as a compulsory public course in the whole school, instead of just limiting to law students.

The article "On the Problems and Countermeasures of College Students' Mental Health and Safe Work under Network Environment" was retracted in 2023. Reasons: signs of a paper mill; suspected computer-generated content; unreliable results or conclusions; concerns about the data.

Second, the daily practice of network laws and regulations is strengthened, so that students abide by the law and use it. On the basis of mastering certain knowledge of network law, college students should consciously abide by network laws and regulations in their daily network environment activities, conscientiously fulfill their responsibilities and obligations in cyberspace, and be strict abiders of network laws and regulations. In the face of infringement of rights and campus safety, college students should learn to use network laws and regulations to protect their rights and interests.

### 4.5. Emphasize Moral Education and Improve Self-Discipline

The governance and construction of cyberspace require the mandatory restraint of laws and regulations on the one hand and the flexible restraint of moral codes on the other. Through the development of online moral education, students can regulate their own words and actions on the Internet under the constraints of moral codes and form a good environment on the Internet.

Due to the anonymity and freedom of expression in the network environment, the moral norms in the real society become less and less binding on the network. At this time, it is especially important to strengthen college students' online moral education and cultivate students' online self-discipline consciousness and self-control ability. College students' online moral education focuses on cultivating their moral self-discipline consciousness characterized by “prudence.” Educators should appropriately increase the content of network ethics education in the teaching process or specially open a course related to network ethics education, so as to give college students systematic knowledge explanation and theoretical education and make students clear the network ethics requirements they should abide by when participating in network life. The purpose of strengthening online ethics education is to cultivate students' green online behavior, form self-control consciousness and self-discipline ability online, resist the erosion of bad information on the Internet, and promote students' healthy and comprehensive growth.

## 5. Conclusion

With the continuous popularization of Internet technology, the network environment becomes more and more complex. Today's college students are faced with the network environment supported by the Internet and linked by information resources. The network not only changes college students' life and learning style but also changes their cognition of network security and brings about a series of troubles. The influence of network environment on college students' mental health is multifaceted and omnidirectional. All kinds of bad information are full of network space, as college educators fully understand the importance of college students' safety. Colleges and universities should face up to the problems of weak consciousness, weak coping ability, and imperfect teaching system of college students in network security. This paper analyzes the problems and causes of college students' mental health and safety through questionnaire survey and takes targeted measures to better solve the problems of college students' mental health and improve college students' network security ability, so as to ensure the high quality of college students' mental health and safety work under the network environment. The next step will be to strengthen theoretical knowledge, ask more profound questions and ideas, and also analyze the questionnaire data more thoroughly.

The article "On the Problems and Countermeasures of College Students' Mental Health and Safe Work under Network Environment" was retracted in 2023. Reasons: signs of a paper mill; suspected computer-generated content; unreliable results or conclusions; concerns about the data.

## Figures and Tables

**Figure 1:** Survey specific results for registered new account privacy protection.

**Figure 2:** The privacy policy carefully read to investigate the specific results.

**Figure 3:** Events done to investigate the specific results.

**Figure 4:** Handling of the specific results of Internet fraud investigations.

**Figure 5:** Use of network security software to investigate specific results.

**Figure 6:** Proficiency in network security software to investigate specific results.

**Figure 7:** Survey specific results for discount to scanning QR code.

**Figure 8:** Used bank card to access the website provided by the other party.

**Figure 9:** Specific results of the Internet self-control ability survey.

**Figure 10:** Specific results of the survey on the lack of empathy in educational content.

**Figure 11:** Specific results of the network safety education survey.

## Data Availability

The dataset used to support the findings of this study is available from the corresponding author upon request.
